# miR-590-5p Targets Skp2 to Inhibit the Growth and Invasion of Malignant Melanoma Cells

**DOI:** 10.1155/2022/8723725

**Published:** 2022-07-07

**Authors:** Yang Tong, Lei Jin

**Affiliations:** ^1^Department of Plastic, Reconstructive and Aesthetic Surgery, Southwest Hospital Affiliated to the Army Military Medical University, Chongqing 400038, China; ^2^Medical College of Soochow University, Suzhou, Jiangsu, China 215123; ^3^Department of Orthopaedics, Wuxi Hongqiao Hospital, Wuxi, Jiangsu, China 214026

## Abstract

Skp2 participates in the regulation of cell growth cycle and promotes the growth of tumor cells. It was speculated that miR-590-5p could regulate the expression of Skp2 and have therapeutic effects on malignant melanin. In this study, the expression of Skp2 was detected by qRT-PCR and Western blot (WB), and the targeted binding between miR-590-5p and Skp2 was verified by dual luciferase reporting assay. Subsequently, cell proliferation activity was detected by CCK8, cell invasion was detected by Transwell, and cell apoptosis was detected by mitochondrial membrane potential assay. The results indicate that Skp2 is highly expressed in melanoma cells and inhibits the proliferation and invasion of melanoma cells. However, miR-590-5p can bind to Skp2 in a targeted manner. miR-590-5p is underexpressed in melanoma cells, and its overexpression can inhibit Skp2 expression and proliferation and invasion of melanoma cells. Our results showed that miR-590-5p could inhibit melanoma cell development by targeting Skp2. This study provides more therapeutic targets for the treatment of melanoma.

## 1. Introduction

Malignant melanoma (MM) is an aggressive melanoma skin cancer and is extremely aggressive. Although the incidence of melanoma is not high, accounting for about 4%-5% of skin malignancies [1], it has a rapid growth rate and easy to metastases, and the survival rate of patients with metastases is extremely low [2]. So malignant melanoma caused people's extensive attention. Some scholars have found that the incidence of malignant melanoma may be related to ultraviolet radiation, heredity, and the number of melanocytic nevus, and the incidence tends to increase with the increase of age [3, 4]. Surgical resection is the preferred treatment for early malignant melanoma, but if the tumor cells metastasize or infiltrate vital organs, surgical treatment cannot be performed [5]. Therefore, the treatment of melanoma is selected according to the state of an illness. In recent years, due to the research on gene mutation targets of malignant melanoma by domestic and foreign scholars, new molecular targeted therapy drugs have been introduced successively, which improves the survival time of advanced patients and brings hope for survival for patients [6].

S-phase kinase-associated protein 2 (Skp2) acts as an E3 ligase, and its Fbox domain can form SCF (skp1-cullin-F-box) complex with Skp1, Cullin1, and Rbx1 [7]. Skp2, as the E3 ligase of the SCF complex, regulates important cellular biological processes by recognizing substrates for ubiquitination and then degrades phosphorylated P27^Kip1^ via protein-ubiquitin pathway or enhances interactions with other proteins and regulates protein activity, such as cell cycle, DNA repair, Akt activation, and mitosis [8, 9]. For example, the SCF-Skp2 complex regulates the cell cycle by inhibiting degradation of p21^Cip1/Waf1^ and p27^Kip1^ by ubiquitin-mediated cyclin-dependent kinase (CDK) [10]. The stability of cell cycle is an important indicator that a tumor can maintain its continuous proliferation. Previous literature has shown that Skp2 is closely related to the development of tumor cells [11–13]. In melanoma cells, Skp2 has been shown to increase expression in melanoma cells, affecting patient survival [14]. Meanwhile, targeted inhibition of Skp2 has been proved to inhibit the progression of uveal melanoma by inhibiting the ubiquitination of P27 [15]. Therefore, targeted inhibition of Skp2 expression can regulate the proliferation of melanoma, which can be used as a new idea for the treatment of melanoma.

According to literature reports, miRNA regulates the expression of protooncogenes and tumor suppressor genes and plays an important role in tumor therapy [16]. Articles on the role of miRNA in tumor cells also emerge in an endless stream, and relevant studies are mainly focused on breast cancer, lung tumor, liver cancer, prostate cancer, and other cancer cells [17, 18]. Through TargetScan sequence alignment, we found that miR-590-5p had binding sites with Skp2, suggesting that Skp2 is a potential target of miR-590-5p. miR-590-5p is abnormally expressed in a variety of tumor cells and participates in tumor development and also has an inhibitory effect on the cell invasion of melanoma cells [19–21]. We hypothesized that the role of Skp2 in melanoma cells may be regulated by miR-590-5p. Therefore, this study combined genes with miRNA to explore the effects of Skp2 and miR-590-5p on melanoma cells and the mechanism of Skp2 action.

## 2. Materials and Methods

### 2.1. Cell Culture

The melanoma cell lines A375, A875, A2058, and SK-Mel-28 and human normal melanin cell line PIG1 which are used in this study were all derived from Wuxi Hongqiao Hospital. The cells were added into 5 mL medium, mixed evenly, and cultured overnight in a 5% CO_2_ incubator at 37°C. On the second day, the culture medium was replaced and the culture was continued until cell adherence occurred. Discard the supernatant, add EDTA for digestion for 1-2 min, and shake the culture flask to disperse the cells. Centrifuge the cells for 8 min, discard the supernatant, add 2 mL maintenance medium, and disperse the cells with a pipette. The cell suspension was diluted at a ratio of 1 : 2~5 for subculture. Materials and procedures used in this experiment were approved by the Ethics Committee of Wuxi Hongqiao Hospital.

### 2.2. Cell Transfection

Design and construction of Skp2 interference expression vector siRNA and Skp2 overexpression vector pcDNA3.1/Skp2 were designed and synthesized by Guangzhou Ruibo Company. The cells were cultured in serum-free medium for 24 h, and then, the Lipofectamine 2000 (Invitrogen) and vector plasmids were mixed into the cells for culture. The cells were transfected with Skp2 siRNA and were collected to detect gene silencing efficiency for subsequent experiments. Skp2 interference expression vector sequence is as follows: 5′-CCGGGATAGTGTCATGCTAAAGAATCTCGAGATTCTTTAGCATGACACTATCTTTTTG-3′. Skp2 overexpression vector sequence is as follows: 5′-CCGGGCCTAAGCTAAATCGAGAGAACTGAGTTCTCTCGATTTAGCTTAGGCTTTTTG-3′.

### 2.3. qRT-PCR

The cells to be tested were inoculated into 6-well plates. Total RNA of the cells was extracted with TRIzol reagent (Sigma-Aldrich). CDNA was synthesized using RNA reverse transcription kit (ThermoFisher). Finally, using cDNA as template, the target gene was amplified by RT-PCR kit (Sigma-Aldrich). The temperature system is as follows: 94°C 45 s, 56°C 30s, 72°C 30s, 30 cycles, and at last 72°C extension for 10 min. MRNA levels of specific genes were detected by quantitative PCR instrument, and 3 multiple holes were set for miRNA detection of each sample to reduce errors.

### 2.4. Western Blot

The cells were added into 400 *μ*L lysate containing PMSF and placed on ice for cracking for 30 min. Centrifuge at 4°C for 5 min; the supernatant was collected and added to 1 × SDS loading buffer. SDS-PAGE was used for electrophoresis, followed by constant pressure transfer membrane with nitrocellulose membrane. The membrane was transferred into the sealing solution and sealed for 1 h. Anti-rabbit Skp2 antibody (1 : 1000) and anti-rabbit caspase-3 antibody (1 : 2000) (Abcam) were added and incubated at 4°C overnight. On the second day, HRP-labeled secondary antibodies (1 : 10000, Abcam) were added and incubated for 2 h. PBS was washed for three times, developer solution was added for develop color, and images were collected with the *β*-actin as internal reference.

### 2.5. Immunohistochemistry

The paraffin tissue was sectioned and baked at 60°C for 1 h. The slices were dewaxed and hydrated and then placed into 400 *μ*L 30% H_2_O_2_ for 30 min. Then, the slices was immersed in citric acid buffer and microwave repair antigen. The cell sections were added with rabbit anti-Skp2 polyclonal antibody (Abcam, 1 : 500) and incubated overnight. Secondary antibody was added (Abcam) and incubated for 1 h. The slices were added with DAB chromogenic agent and reacted at room temperature for 5 min, and then, hematoxylin was added for redyeing for 2 min; at last, rinse with running water. It was dehydrated with gradient alcohol, sealed with gum, and observed under a microscope.

### 2.6. CCK8

Cells at logarithmic growth stage were taken inoculated into culture plates with 3 multiple wells in each group and cultured for 12, 24, and 48 h. CCK-8 solution (GlpBio) was added into the cells for 2 h, and the absorbance of the cells was determined.

### 2.7. Transwell

The cells were digested with trypsin, cell suspension was added to upper chamber of Transwell, and cell culture medium was added into the lower chamber, and the culture was continued for 24 h. Remove the upper chamber, discard the supernatant that in the upper chamber, and wash with PBS for 3 times. The cells in the upper chamber were fixed in paraformaldehyde and then stained with 0.1% crystal violet solution. The migrating cells were observed using a microscope.

### 2.8. Double Luciferase Reporter Gene Assay

The complementary binding sites of miR-590-5p and Skp2 were predicted using TargetScan software. We structured the Skp2-wt/mut luciferase reporter vector plasmids. The luciferase reporter vector plasmids were transfected into HEK-293T cells, respectively, and the cells were incubated in an incubator for 20 min. Double luciferase reporter gene assay kit (Yesen Biotechnology Co., Ltd.) was used to detect the luciferase activity in the cells.

### 2.9. Colony Formation Assays

The cells were dispersed by adding 0.25% trypsin and added to DMEM medium containing 10% fetal bovine serum to prepare cell suspension. The cells were inoculated in Petri dishes at 100 per dish. The Petri dishes were placed in an incubator with 5% CO_2_ at 37°C for 1-2 weeks. When obvious cell clones appeared in Petri dish, wash it with PBS twice carefully. The cells were fixed in 4% paraformaldehyde for 15 min. Using a microscope, watch the cells grow and count them.

### 2.10. Mitochondrial Membrane Potential Detection

Mitochondrial membrane potential detection kit (Leagene Biotechnology Co., Ltd., Beijing) was used to detect cell apoptosis rate. First, JC-1 working fluid was prepared according to the instructions. The cells were collected, cleaned with PBS solution, and centrifuged to discard supernatant. The precipitates were suspended in 0.5 mL culture medium containing serum and phenolic erythrocytes. The culture medium was mixed with 0.5 mL JC-1 staining solution and placed in incubator for incubation at 37°C for 20 min. The culture medium was centrifuged at 4°C for 5 min, and the precipitation was washed twice with diluted JC-1 Buffer (1×) and suspended again. Cell apoptosis was observed using fluorescence microscopy.

### 2.11. Statistical Analyses

SPSS 20.0 statistical software was used to calculate and process the experimental data. The measurement data in the experiment are mainly expressed as mean ± standard deviation. Comparison between groups was performed by *t* test. All experiments were repeated more than 3 times.

## 3. Results

### 3.1. Skp2 Expression in Malignant Melanoma Cells

First, we examined Skp2 expression level in malignant melanoma. Skp2 was highly expressed in both malignant melanoma cells and tissues, as opposed to normal tissue cells (Figures 1(a) and 1(b)). The expression level of Skp2 in different malignant melanoma cell lines was higher than that in normal melanocytes (Figure 1(c)). Subsequently, immunohistochemical results showed that Skp2 was significantly expressed in melanoma nuclei (Figure 1(d)). The Skp2 expression is upregulated in melanoma cells and tissues, suggesting that Skp2 may be involved in the development of malignant melanoma cells.

### 3.2. Effects of Skp2 on Proliferation and Invasion of Melanoma Cells

Previous literature have shown that Skp2 expression is upregulated in multiple cancer cells, so we transfected Skp2 siRNA into melanoma cells to knock down Skp2 expression. The results showed that Skp2 expression in the Skp2 siRNA group decreased, and siRNA was successfully transfected (Figure 2(a)). Subsequently, the cell proliferation and invasion were reduced after transfection with Skp2 siRNA (Figures 2(b) and 2(c)). Skp2 expression can promote the growth and invasion of melanoma cells.

### 3.3. miR-590-5p Targeted Binding Skp2

The binding sequence of Skp2 to miR-590-5p was analyzed by website (Figure 3(a)). qRT-RCP detection showed that miR-590-5p expression was low in all malignant melanoma cells (Figure 3(b)). The results of the double luciferase report showed that luciferase activity was decreased in miR-590-5p mimics+Skp2-wt group (Figure 3(c)). Subsequently, we found that miR-590-5p could negatively regulate Skp2 expression (Figures 3(d) and 3(e)). Therefore, miR-590-5p can regulate Skp2 expression and is negatively correlated with Skp2 expression.

### 3.4. miR-590-5p Targets Skp2 to Inhibit the Growth and Proliferation of Melanoma Cells

Then, the role of miR-590-5p in melanoma cells was studied. According to the qRT-PCR results, the expression of miR-590-5p in melanoma cells was lower than that in normal epithelial cells (Figure 4(a)). However, the high expression of miR-590-5p significantly reduced the proliferation and invasion ability of cells (Figures 4(b) and 4(c)). Therefore, combined with the above studies, upregulation of miR-590-5p expression can target Skp2 expression and inhibit cell proliferation and invasion.

### 3.5. Overexpression of Skp2 Partially Reversed the Inhibition of miR-590-5p

To further prove this point, we transfected Skp2 overexpression vector pcDNA3.1/Skp2 into A375 cells. The result shows that Skp2 expression was decreased and caspase-3 expression was increased after the cell transfection with miR-590-5p mimics. After increased Skp2 expression, Skp2 expression was increased and apoptosis factor caspase-3 expression was significantly decreased compared with miR-590-5p mimics (Figure 5(a)).

Continue to study the ability of cells to proliferate and apoptosis. We found that miR-590-5p inhibited the cell colony formation rate. When Skp2 expression was increased, the colony formation rate was significantly increased (Figure 5(b)). Apoptosis was then detected using mitochondrial membrane potential. The mitochondria fluorescence was decreased and cell apoptosis was increased in miR-590-5p mimic group, while mitochondria fluorescence was increased and cell apoptosis was decreased after cotransfection with pcDNA3.1/Skp2 (Figure 5(c)). Therefore, Skp2 overexpression can partially reverse the inhibitory effect of miR-590-5p, again verifying the targeting relationship between miR-590-5p and Skp2.

## 4. Discussion

Skp2 is involved in the development of several tumor cells, such as lymphoma, prostate cancer, pancreatic cancer, breast cancer, nasopharyngeal cancer, and gastric cancer [22]. Therefore, Skp2 could promote tumor cell proliferation and invasion in tumor cells, mainly acting as an oncogene. For example, dysregulation of Skp2 expression plays a carcinogenic role in hematological malignancies [23]. The overexpression of Skp2 in retinoblastoma can restore suppressed retinoblastoma growth [24]. Therefore, many experts and scholars are using Skp2 as a target for cancer treatment to explore more cancer treatment methods. For example, inhibition of Skp2 expression can sensitize chronic myeloid leukemia cells to imatinib and induce cell apoptosis. The result of treatment of synovial sarcoma cells was with Skp2 inhibitor flavokawain A (FKA) showing that Skp2 inhibitor can induce cell growth cycle arrest [25, 26]. Inhibition of Skp2 expression can effectively lead to growth cycle arrest of cancer cells and induce apoptosis.

miR-590-5p plays an anticancer miRNA role in multiple tumor cells. For example, miR-590-5p can be involved in regulating the development of tongue squamous cell carcinoma or can regulate the apoptosis of heart failure cells [27, 28]. miR-590-5p also has a certain effect on the treatment of cardiovascular diseases [29]. There are still many studies on the therapeutic effects of miR-590-5p.

In this study, we found that both miR-590-5p and Skp2 were abnormally expressed in melanoma cells. This suggests that both miR-590-5p and Skp2 are involved in the treatment of malignant melanoma. Inhibition of Skp2 expression can effectively inhibit the proliferation and invasion of melanoma cells. This study also confirmed the specific binding between miR-590-5p and Skp2. miR-590-5p inhibits Skp2 expression and inhibits melanoma cell development, while overexpression of Skp2 could reverse the inhibitory effect of miR-590-5p. This results further demonstrated the therapeutic effect of miR-590-5p on melanoma cells. However, this study still has shortcomings. It is known in this study that miR-590-5p can regulate Skp2 function, but the downstream pathway of Skp2 is not clear, and further research is needed in the future.

## 5. Conclusion

In this study, we found that miR-590-5p can inhibit the proliferation of melanoma cells and induce their apoptosis by targeting Skp2 expression. The results of this study provide new targets and genes for the treatment of melanoma. Skp2 is also abnormally expressed in uveal melanoma, and more and more effective treatments can be explored based on miR-590-5p and Skp2 in the future.

## Figures and Tables

**Figure 1:** Expression of Skp2 in malignant melanoma cells. (a and b) qRT-PCR was used to detect the expression of Skp2 mRNA in melanoma cells and tissues. (c) The expression of Skp2 protein was detected using WB. (d) The expression of Skp2 protein was detected by IHC. Compared to the control group, ^∗^*P* < 0.05.

**Figure 2:** Effect of Skp2 expression on proliferation and invasion of melanoma cells. Cells were transfected with Skp2 siRNA. (a) The Skp2 protein expression was detected. (b) Cell proliferation ability was detected. (c) Transwell was used to detect cell invasion. Compared to the control group, ^∗^*P* < 0.05.

**Figure 3:** Targeted binding of miR-590-5p to Skp2. (a) Sequence analysis of binding sites. (b) qRT-PCR was used to detect the expression of miR-590-5p in different melanoma cell lines. (c) Luciferase activity was detected. (d and e) The expression of Skp2 mRNA and protein was detected. Compared to the control group, ^∗^*P* < 0.05.

**Figure 4:** Effects of miR-590-5p on the growth and proliferation of melanoma cells. (a) The expression of miR-590-5p mRNA was detected. (b) CCK8 was used to detect cell proliferation. (c) Transwell was used to detect cell invasion. Compared to the control group, ^∗^*P* < 0.05.

**Figure 5:** Effect of miR-590-5p targeting Skp2 on proliferation and invasion of melanoma cells. Cotransfection of miR-590-5p and Skp2 overexpression vector. (a) The expression of Skp2 and caspase-3 was detected using WB. (b) The colony formation ability of cells was detected. (c) The changes of mitochondrial membrane potential were detected. Compared to the control group, ^∗^*P* < 0.05; compared to the miR-590-5p mimic group, ^#^*P* < 0.05.

## Data Availability

The data used to support the findings of this study are included within the article.
